# Pancreatic Cancer Cell Glycosylation Regulates Cell Adhesion and Invasion through the Modulation of α2β1 Integrin and E-Cadherin Function

**DOI:** 10.1371/journal.pone.0098595

**Published:** 2014-05-30

**Authors:** Sònia Bassagañas, Sandra Carvalho, Ana M. Dias, Marta Pérez-Garay, M. Rosa Ortiz, Joan Figueras, Celso A. Reis, Salomé S. Pinho, Rosa Peracaula

**Affiliations:** 1 Biochemistry and Molecular Biology Unit, Department of Biology, University of Girona, Girona, Spain; 2 Institute of Molecular Pathology and Immunology of the University of Porto (IPATIMUP), Porto, Portugal; 3 Department of Pathology, Dr. Josep Trueta University Hospital, Girona, Spain; 4 Department of Surgery, Dr. Josep Trueta University Hospital, IdIBGi, Girona, Spain; 5 Institute of Biomedical Sciences of Abel Salazar (ICBAS), University of Porto, Porto, Portugal; 6 Medical Faculty, University of Porto, Porto, Portugal; INRS, Canada

## Abstract

In our previous studies we have described that ST3Gal III transfected pancreatic adenocarcinoma Capan-1 and MDAPanc-28 cells show increased membrane expression levels of sialyl-Lewis x (SLe^x^) along with a concomitant decrease in α2,6-sialic acid compared to control cells. Here we have addressed the role of this glycosylation pattern in the functional properties of two glycoproteins involved in the processes of cancer cell invasion and migration, α2β1 integrin, the main receptor for type 1 collagen, and E-cadherin, responsible for cell-cell contacts and whose deregulation determines cell invasive capabilities. Our results demonstrate that ST3Gal III transfectants showed reduced cell-cell aggregation and increased invasive capacities. ST3Gal III transfected Capan-1 cells exhibited higher SLe^x^ and lower α2,6-sialic acid content on the glycans of their α2β1 integrin molecules. As a consequence, higher phosphorylation of focal adhesion kinase tyrosine 397, which is recognized as one of the first steps of integrin-derived signaling pathways, was observed in these cells upon adhesion to type 1 collagen. This molecular mechanism underlies the increased migration through collagen of these cells. In addition, the pancreatic adenocarcinoma cell lines as well as human pancreatic tumor tissues showed colocalization of SLe^x^ and E-cadherin, which was higher in the ST3Gal III transfectants. In conclusion, changes in the sialylation pattern of α2β1 integrin and E-cadherin appear to influence the functional role of these two glycoproteins supporting the role of these glycans as an underlying mechanism regulating pancreatic cancer cell adhesion and invasion.

## Introduction

Cell adhesion is a dynamic process that allows cells of multicellular organisms to be cohesive, communicate and interact among them and with the extracellular matrix (ECM), playing an essential role in many cellular functions, such as cell normal embryonic development, morphogenesis and tissue repair, as well as in many pathological processes such as tumor invasion and metastasis, thrombosis and inflammation [1]. Cancer invasion is an heterogeneous process for which the physical, cellular and molecular determinants adapt and react throughout the progression of the disease in a cell- and tissue-driven manner [2]. A key stone of cancer invasion is the disruption of the cellular junctions through the downregulation of the function and/or important signaling pathways carried out by critical cell adhesion molecules (CAMs) such as cadherins and integrins. This loss of adhesiveness allows tumor cells to disobey the social order, resulting in the alteration of the normal histological structure and dissociation from cancer nests [3].

In particular, *adherens junctions* (AJ), which are orchestrated by E-cadherin molecule, provide adhesive contacts between neighboring epithelial cells and form intracellular interactions to the actin cytoskeleton, being involved in important signaling processes leading to the regulation of gene transcription [4], [5]. It is not surprising that in most, if not all, cancers of epithelial origin E-cadherin-mediated cell-cell adhesion is downregulated or inactivated promoting cancer cell invasion and metastases. In addition, E-cadherin is one of the key molecular markers along the process of Epithelial to Mesenchymal Transition (EMT), which is a fundamental biological process associated with the progression from adenoma to carcinoma and the subsequent steps of cancer cell invasion and metastasis [6], [7].

Integrins are transmembrane receptors that bind to ECM components and are involved in adhesion and migration processes. They are composed of α and β heterodimers, lack endogenous enzymatic activity and depend on signal transducers to perform their functions, such as the nonreceptor focal adhesion kinase (FAK) as well as a variety of scaffolding proteins that link integrins to the actin cytoskeleton [8]. As a result of cell adhesion to ECM components, integrins transmit information that regulates intracellular signaling. Specifically, FAK is activated via autophosphorylation at tyrosine 397 (Y397) upon integrin binding to its ligands. Phosphorylated FAK Y397 becomes a binding site for the tyrosine kinase Src, and FAK/Src complex then activates other downstream proteins, e.g. pCAS, Crk or paxillin, which in turn activate important pathways involved in cell migration progress [9].

Pancreatic ductal adenocarcinoma (PDAC) is the fourth leading cause of cancer death, with a 5-year survival rate of less than 5%. This extremely poor outcome is mainly due to its aggressiveness and delay in diagnosis, since approximately 85% of patients are diagnosed at advanced stages of disease, when metastasis is already present [10]. Therefore, there is an urgent need to identify the underlying molecular mechanisms of PDAC, envisioning potential clinical applications.

PDAC is characterized by an intense desmoplastic response, suggesting a role for ECM cell adhesion molecules, such as integrins, throughout the tumorigenic process [11], [12]. A number of reports have described the up-regulation and delocalization of several integrin subunits, including α1, α2, α3 and α6 subunits in pancreatic cancer [13], [14]. Furthermore, β1 integrins have been reported to play an essential role in promoting adhesion and invasion of pancreatic carcinoma and, in the case of α2β1 integrin, in mediating the malignant phenotype on type 1 collagen in pancreatic cancer cell lines [15], [16].

On the other hand, downregulation or inactivation of E-cadherin expression has also been associated with poor survival and acquisition of invasiveness, as well as dedifferentiation of PDAC [17].

Glycosylation is one of the most important protein post-translational modification and tumor cells frequently display an altered pattern of cell surface glycosylation in relation to their normal counterparts, which directly influences several cellular processes, including cell-cell adhesion [18] and cell-ECM interaction [19], [20]. In particular, several pancreatic adenocarcinoma cells have been described to exhibit an increase in the expression of the Lewis-type sialylated epitopes sialyl-Lewis a (SLe^a^) and sialyl-Lewis x (SLe^x^) and the correspondent glycosyltransferases involved in their biosynthesis, which have been correlated with PDAC invasiveness and metastasis [21], [22], [23], [24].

Furthermore, several studies have reported that *N*-glycans influence the stability of AJ and E-cadherin biological functions in a variety of tumors [25], [26], [27]. In addition, integrins are also carriers of *N*-glycans, and changes in glycan branching and sialylation of integrins have been reported to influence integrin binding to ECM and cell migration capabilities although the mechanisms underlying these actions are still unknown [28], [29].

In previous studies we have described that α2,3-sialyltransferase ST3Gal III transfection of pancreatic adenocarcinoma cell lines Capan-1 and MDAPanc-28 leads to the overexpression of SLe^x^ antigen and the decrease of α2,6-sialic acid in their cell surface. ST3Gal III transfectants exhibited loss of cell-ECM adhesion, increased motility rates through type 1 collagen and an enhanced metastatic phenotype *in vivo* [23], [30]. To understand this enhanced metastatic phenotype *in vivo*, we here address whether cell-cell adhesiveness and cell invasion are also affected by the cell sialylation changes using the stably transfected cell line models. We have also determined whether the cell surface glycan differences between transfected and control cells could be displayed in their α2β1 integrin and E-cadherin molecules and could thus modulate their function.

## Materials and Methods

### Ethics statement

The use of specimens from human subjects was approved by the Ethics Committee of Dr. Josep Trueta University Hospital from Girona (Spain).

### Cell culture

Human pancreatic adenocarcinoma cell lines Capan-1 (ATCC n°HTB-79; MD, USA) and MDAPanc-28, and the described stable ST3Gal III transfected (C31 and M34, respectively) and mock transfected (CP and MP, respectively) [23], [30] were used in this work. Cells were cultured in Dulbecco's Modified Eagle's Medium (DMEM) GlutaMAX-I containing 10% Fetal Bovine Serum (FBS), 100 U/mL Penicillin G, 100 mg/mL Streptomycin, 0.25 mg/mL Amphotericin B, and supplemented with 400 µg/ml (Capan-1 transfectants) or 800 µg/ml (MDAPanc-28 transfectants) Geneticine G-418 (all of them from Gibco, UK), under a humidified atmosphere containing 5% CO_2_. For the experiments, 3.5×10^5^ Capan-1/CP/C31 or 5.5×10^5^ MDAPanc-28/MP/M34 cells were seeded in 75 cm^2^ flasks (Nunc, Roskilde, Denmark) and cultured for 84 h (exponential growth).

### Flow cytometry analysis

Detection of integrin subunits and E-cadherin was performed by indirect immunofluorescence. Cells (5×10^5^) were incubated at 4°C for 30 min in the presence or absence of monoclonal antibodies (mAb) against integrin subunits β1 (clone TDM29, Chemicon, CA, USA; diluted 1/10), α2 (clone P1E6, Chemicon; 1/200) or mAb against human E-cadherin (clone HECD-1, Zymed Labs CA, USA; 1/50). After a wash, cells were incubated with the secondary antibody Alexa Fluor 488 goat anti-mouse IgG (Invitrogen Life Technologies, MD, USA). Antibodies were diluted in Phosphate Buffered Saline (PBS) containing 1% Bovine Serum Albumin (BSA). Mean Fluorescence Intensity (MFI) was calculated as the quotient between the positive and negative GeoMean for each cell line. For each sample three independent assays were performed.

### Cell adhesion assay to collagen

Cell adhesion assays were performed as previously described [30]. 96-well microplates were coated with a solution of 10 µg/ml type 1 collagen from calf skin (Sigma-Aldrich; MO, USA) in PBS, or PBS-1% BSA. For each well, 2.5×10^4^ cells were seeded and incubated at 37°C for 20 min. In selected experiments, cells were previously incubated with function-blocking mAbs against integrin subunits α2 (clone P1E6, Chemicon; 1/50 in PBS), α3 (clone P1B5, Calbiochem, CA, USA; 1/50), α5 (clone P1D6, Chemicon; 1/50) or β1 (clone TDM29, Chemicon; 1/5) for 30 min at 4°C. After three washes, adherent cells were estimated with the MTT method (Sigma). Three independent experiments were performed in quadruplicate. Results were expressed as the mean ± standard deviation (SD) of values of specific binding to type 1 collagen (OD 570 nm of cells bound – OD 570 nm of cells bound to PBS-1% BSA).

### Type 1 collagen migration assay

Cell migration was evaluated using modified Boyden chambers as previously described [23], [30]. Briefly, serum starved cells were detached, resuspended in serum-free medium and seeded onto type 1 collagen coated inserts (Greiner Bio-One GmbH; Austria) containing DMEM-1% FBS. In selected experiments, cells were previously incubated with function-blocking mAbs against α2 (clone P1E6, Chemicon; diluted 1/50 in PBS) or β1 (clone TDM29, Chemicon; 1/5) integrin subunits. After 8 h, non-migrated cells were wiped from the top surface of the filter and migrated cells were fixed, stained with hematoxylin-eosin and counted. Results were expressed as the average number of migrated cells per well ± SD, obtained from two separate experiments performed in duplicate.

### Matrigel invasion assay

Matrigel invasion was performed following described procedures [31]. 24-well Matrigel-coated invasion inserts (BioCoat Matrigel Invasion Chambers; BD Biosciences, CA, USA) were rehydrated with DMEM-10% FBS for 1 h at 37°C. Cells (5×10^4^) were seeded onto the coated inserts and incubated for 24 h in standard conditions. Non-invasive cells were carefully wiped from the top surface of the filter and invasive cells were fixed with ethanol and stained with Vectashield mounting medium with DAPI (Vector Laboratories, CA, USA). Results were expressed as the average number of invasive cells per well ± SD obtained from two separate experiments performed in duplicate.

### Slow aggregation assay

Slow aggregation assay on agar was based on a previously described method [32]. 96-well plates were coated with 50 µl of semi-solid agar medium consisting of 100 mg agar (Bacto Agar, BD Biosciences) in 15 ml distilled water and sterilized through boiling three times for 10 s. After jellification, a single-cell suspension of 2×10^4^ cells was seeded onto the agar. Cell aggregation was evaluated after 24 h and particle size was measured in pixels using ImageJ 1.42q software.

### Western blot and lectin blot analysis of total cell lysates

Cells were washed with cold PBS and resuspended in lysis buffer containing 1% (v/v) Triton X-100, 1% (v/v) NP-40, protease inhibitor cocktail (Roche Diagnostics, Indianapolis, USA), 100 mM Na_3_VO_4_ and 100 mM PMSF in PBS, for 15 min on ice. The protein content of the total cell lysates (TCL) was quantified by bicinchoninic acid (BCA) assay kit (Pierce, IL, USA) and afterwards the overall expression of sialic acids and E-cadherin was evaluated with 50 µg or 20 µg, respectively. Samples were resuspended in Laemmli buffer and heated to 96°C for 5 min. Lysates were subjected to a 7.5% SDS-PAGE and transferred onto a nitrocellulose membrane. After blocking with PBS-5% BSA containing 0.05% Tween 20 (PBST) (for sialic acids blot) or 5% low-fat milk in PBS containing 0.01% Tween 20 (for E-cadherin blot), membranes were incubated with mAb against SLe^x^ (clone KM93, Calbiochem; 1/100) or E-cadherin (clone 36, BD Biosciences; 1/3000) in PBST-5% low-fat milk overnight at 4°C; or with biotynilated *Sambucus nigra* agglutinin (SNA) or biotynilated *Maackia amurensis* lectin II (MAL-II) (Vector Laboratories) diluted 1/200 in PBST-1% BSA for 1 h at room temperature. Membranes were washed and incubated with the secondary antibody HRP (horseradish peroxidase)-conjugated rabbit anti-mouse IgM (Santa Cruz Biotechnology; CA, USA) to detect SLe^x^, HRP-conjugated goat anti-mouse (Santa Cruz) to detect E-cadherin or Vectastain Elite ABC kit (Vector Laboratories) to detect sialic acids. For loading control analysis, mouse antibody against human tubulin (Sigma; diluted 1/10000 in PBST), and secondary antibody HRP-conjugated goat anti-mouse (Santa Cruz) were used. Immunoreactive bands were visualized using ECL Reagent (GE Healthcare, NJ, USA). At least three independent experiments were performed.

### E-cadherin immunoprecipitation

For E- cadherin immunoprecipitation, 750 µg of TCL were precleared with 25 µl of protein G-sepharose beads (GE Healthcare) for 1 h at 4°C, as previously described [33]. Briefly, after centrifugation the supernatants were incubated overnight with 2.5 µg of mAb against human E-cadherin (clone 36, BD Biosciences), and after that the immune complexes were released by boiling and subjected to 7.5% SDS-PAGE. Western blot and lectin blot analyses were performed as described above. Three independent experiments were undertaken.

### Cell surface biotinylation, cell lysis and α2β1 immunoprecipitation

Cell surface biotinylation was performed following described procedures [34] with minor modifications. Exponential CP and C31 cells were detached, washed three times with ice-cold PBS and incubated with 1 mg/ml sulfo-NHS-LC-biotin (Sigma) in PBS for 25 min at room temperature on a rocking platform. After incubation, three washes with PBS-100 mM glycine were carried out to quench any unreacted biotinylation reagent. Cells were lysed by incubation with lysis buffer [50 mM Tris-HCl pH 7.5, 150 mM NaCl, 1% (v/v) Triton X-100, 10 µg/ml leupeptin, 20 µg/ml aprotinin, 5 mM PMSF, 1 mM benzamidine hydrochloride hydrate, 10 mM MgCl_2_ and 10 mM EGTA]. Lysates were cleared by centrifugation, supernatants were collected and protein content was determined by Bradford (Biorad). For α2 integrin immunoprecipitation, 50 µl of protein A sepharose CL-4B beads (GE Healthcare) were incubated with 0.5 µl of rabbit polyclonal antibody against α2 integrin (Chemicon) for 2 h at 4°C on a rocking platform. Afterwards, 400 µg of protein sample were incubated with the protein A-antibody complexes overnight at 4°C on the rocking platform. Beads were collected by rapid centrifugation and washed three times with washing buffer [50 mM Tris-HCl pH 7.5, 150 mM NaCl, 0.1% (v/v) Triton X-100, 1 mM MgCl_2_ and 10 mM EGTA].

### Western blot and lectin blot analysis of the integrin immunoprecipitates

Immunoprecipitates were resuspended in reducing buffer and heated to 100°C for 6 min. Then, they were loaded and resolved on an 8% SDS-PAGE, and transferred to a PVDF membrane. The blots were probed with mAb against SLe^x^ [clone KM93, Calbiochem; diluted 1/67 in TBST buffer (Tris-HCl 10 mM pH 7.5, NaCl 100 mM, 0.1% Tween 20) containing 0.5% BSA)]; or with fluorescein conjugated SNA lectin [Vector Laboratories; diluted 1/1000 in lectin buffer (150 mM NaCl, 0.1 M Tris-HCl pH 7.5, 1 mM CaCl_2_, 1 mM MgCl_2_, 1 mM MnCl_2_)] for 2 h at room temperature. After three washes with TBST, membranes were incubated with secondary antibody HRP-conjugated goat anti-mouse (Abcam, UK; diluted 1/40000 in TBST-0.5% BSA); or sheep anti-fluorescein (Roche Diagnostics, diluted 1/2500 in TBST-1% BSA), respectively, for 1 h at room temperature. Immunoreactive bands were visualized using Immobilon Western Chemiluminescent HRP Substrate kit (EMD Millipore Corporation; MA, USA). Equal amounts of loaded α2 integrin were corroborated by stripping the membranes and blotting with HRP-conjugated streptavidin (GE Healthcare; diluted 1/100000 in TBST-1% BSA). Two independent experiments were performed.

### Tyrosine phosphorylation assay of Focal Adhesion Kinase (FAK)

Tyrosine phosphorylation assays of FAK were performed following described procedures [35]. CP and C31 serum-starved cells at exponential growth were detached and held in suspension for 60 min to reduce the detachment-induced activation. To perform this assay, 2×10^5^ cells were plated onto type 1 collagen CELLCOAT 24-well dishes (Greiner Bio-One) or kept in suspension for 20 min at 37°C. After two washes with PBS the cells were lysed by incubation with RIPA B lysis buffer [20 mM phosphate buffer, 1% (v/v) Triton X-100, 150 mM NaCl, 5 mM EDTA, 5 mM PMSF, 1% (v/v) aprotinin, 10 µg/ml leupeptin, 250 µg/ml Na_3_VO_4_]. Lysates were cleared by centrifugation, supernatants were collected and protein content was determined. Then 20-25 µg of protein were resuspended in reducing buffer and heated to 70°C for 15 min. Samples were resolved on an 8% SDS-PAGE, electrophoretically transferred into a PVDF membrane and blotted with mAb against human FAK phosphotyrosine 397 (clone 18, BD Biosciences; diluted 1/1000 in TBST-1% BSA) for 1 h at room temperature. Equal loading was confirmed by blotting with mAb against total human FAK (clone 77, BD Biosciences; 1/500 in TBST-5% non-fat milk). Secondary antibody was HRP-conjugated goat anti-mouse (Abcam; 1/40000 in TBST-0.5% BSA). Immunoreactive bands were visualized as described above. Two independent experiments were undertaken. Relative FAK Y397 phosphorylation per cell line was calculated as the quotient between pY397 FAK quantification and total FAK quantification.

### Immunofluorescent double-labeling of cultured cells

Cells (4×10^4^) were seeded on 24 well plates (Nunc) with coverslips on the bottom of each well and cultured for 24 h, until nearly confluent monolayers. Then cells were washed with PBS, fixed in ice-methanol for 20 min, and blocked with PBS-10% BSA for 30 min. For E-cadherin staining, cells were incubated with mAb against E-cadherin (clone 36, BD Biosciences; 1/200) and with secondary antibody Alexa Fluor 488 goat anti-mouse IgG (Invitrogen Life Technologies, 1/500). For double labeling, cells were incubated with mAb against SLe^x^ (clone KM93, Calbiochem; 1/60) and secondary antibody Alexa Fluor 594 goat anti-mouse IgM (Texas Red-conjugated; Invitrogen Life Technologies; 1/500). Finally, cells were washed, stained with DAPI (Sigma) and mounted with Vectashield mounting medium (Vector Laboratories). Antibodies were diluted in PBS-5% BSA, and incubated in a dark and humid chamber at room temperature. Separate images for E-cadherin, SLe^x^ and DAPI were captured digitally at 40× or 63× magnification. The green (for FITC), red (for Texas Red) and blue (for DAPI) components were merged and combined images were imported into Adobe Photoshop.

### Tissue specimens immunofluorescence

Two control pancreatic tissue samples from healthy donors and five pancreatic adenocarcinoma tissues were obtained from patients undergoing surgical resection. The histopathologic features of the resected specimens were confirmed by the pathologists. These patients included three male and two females ranging 49–72 years with exocrine adenocarcinomas of duct cell type; four were stage IIB (two well differentiated, one moderately differentiated and one poorly differentiated), and one stage IIA (moderately differentiated) according to the Tumor Node Metastasis Classification of Malignant Tumors of the International Union Against Cancer (UICC) 7th edition [36]. Tissues were fixed in 10% formalin, embedded in paraffin and cut into 5 µm serial sections.

For E-cadherin and SLe^x^ immunofluorescence, paraffin sections were dewaxed, rehydrated and treated with Extran 0.05% (Merck, Germany) in distilled water for 15 min in a microwave oven at 750 W. After cooling at room temperature, slides were rinsed twice in PBS and incubated for 20 min with rabbit non-immune serum at a dilution 1/5 in PBS-10% BSA, then incubated with mAb against E-cadherin (clone 36, BD Biosciences, 1/100) overnight at 4°C and afterwards with secondary antibody FITC-conjugated rabbit anti-mouse (Dako, Denmark, 1/100). Then slides were blocked with non-immune goat serum diluted 1/5 in PBS-10% BSA for 20 min, incubated with mAb against SLe^x^ (clone KM93, Calbiochem; 1/60) overnight at 4°C, and finally incubated for 30 minutes with Texas Red-conjugated goat anti-mouse IgM (Jackson Immunoresearch, PA, USA; 1/50). Nuclei were stained with DAPI and slides were mounted with Vectashield mounting medium. Antibodies were diluted in PBS-5% BSA, and incubations were performed in a dark and humid chamber at room temperature. Microscopy images were obtained under fluorescence microscope as described in the above protocol.

For α2β1 integrin and SLe^x^ immunofluorescence, paraffin sections were dewaxed, rehydrated and treated with 10 mM sodium citrate (pH 6) and microwaved on high for 10 min. Next, they were washed three times with PBS (pH 7.4), incubated for 30 min in 0.3 M glycine in PBS for autofluorescence reduction and washed again. Next nonserum protein block (Dako) was applied for 10 min and then removed. After washing three times with PBS, 5% normal goat serum in PBS was applied for 20 min and removed by blotting. Sections were then incubated with primary antibody diluted in 5% normal goat serum (1/20 for mAb against β1 integrin, clone TDM29, Chemicon; and 1/1000 for rabbit polyclonal antibody against α2 integrin, AB1936, Chemicon) for 60 min at room temperature and washed three times in PBS. Afterwards the slides were incubated with FITC-conjugated goat anti-mouse or goat anti-rabbit (Invitrogen Life Technologies) diluted 1/500 in 5% normal goat serum for 30 min, and washed with PBS. Then, slides were incubated with mAb against SLe^x^ (clone KM93, Calbiochem; 1/60) for 60 min, washed with PBS and finally incubated for 30 minutes with Texas Red-conjugated goat anti-mouse IgM (Molecular Probes), diluted 1/500 in normal goat serum. Nuclei were stained with DAPI and slides were mounted with Fluorescent mounting medium (Dako). Immunolabeled preparations were evaluated using a NIKON A1R+ confocal laser scanning microscope as described in the above protocol. For negative controls, preimmune serum instead of primary antibodies was used.

### Statistical analysis

Data were expressed as mean ± SD. Data was normalized using the Kolmogorov-Smirnov test and the homogeneity of variances was checked using the Levene's test. Mean scores were compared with Student's t-test or one-way ANOVA and Tukey's test for multiple comparisons, using SPSS statistical software for Windows (version 15.0, SPSS Inc.; Chicago, IL, USA). The criterion for significance was set at p<0.05.

## Results

### Characterization of SLe^x^ and α2,6-sialic acid content in total cell lysates from ST3Gal III and mock transfected Capan-1 and MDAPanc-28 clones

ST3Gal III transfectants of Capan-1 and MDAPanc-28 have been described to increase cell surface SLe^x^ levels concomitantly with a decrease in α2,6-sialic acid [23]. From the characterized ST3Gal III overexpressing clones (C31 and C32 for Capan-1, and M33 and M34 for MDAPanc-28) that showed similar behavior, the highest ST3Gal III and SLe^x^ expressing clones from each cell line, C31 and M34, were chosen to address the influence of sialylated determinants in cell adhesion and invasion processes, as well as in E-cadherin and α2β1integrin function. They were compared to the control mock clones, CP and MP, respectively.

In order to evaluate the changes in protein glycosylation, the overall SLe^x^ and α2,6-sialic acid content of total cell lysates (TCL) from the four transfected cell lines was analyzed by Western and lectin blot. Higher expression of SLe^x^ was detected in Capan-1 cell model compared to MDAPanc-28 model; conversely, higher expression of α2,6-sialic acid structures was present in the MDAPanc-28 model (**Figure 1**). ST3Gal III transfected clones C31 and M34 showed higher SLe^x^ levels compared to their respective controls, with marked differences in C31 cells (**Figure 1A**). At the same time, a concomitant decrease in the expression of α2,6-sialic acid structures was observed in the ST3Gal III transfected clones compared to the controls (**Figure 1B**), which was more relevant in M34 cells. Arrows in **Figure 1** indicate the protein bands that show increases in SLe^x^ or α2,6-sialic acid levels between the ST3Gal III transfectants and their corresponding mock cells. These results showed a competitive expression between α2,3- and α2,6-sialic acid, which are in accordance with the competition among α2,3-sialyltransferases ST3Gal III-IV and α2,6-sialyltransferase ST6Gal I enzymes to sialylate type II glycan chains previously described [23].

**Figure 1:** SLe^x^ and α2,6-sialic acid determinants content in total cell lysates. SLe^x^ and α2,6-sialic acid content of total cell lysates (TCL) from the transfected cell lines (C31 and M34) and their respective controls (CP and MP) was analyzed by Western and lectin blot. Blots were probed with clone KM93 mAb against SLe^x^ epitope (**A**) or *Sambuccus nigra* agglutinin (SNA), which detects α2,6-sialic acid structures (**B**). Tubulin (50 kDa) was used as loading control in each cell line. Arrows indicate the protein bands that show increases in SLe^x^ or α2,6-sialic acid levels between the ST3Gal III transfectants and their corresponding mock cells.

It is important to notice that the differences in sialic acid content between ST3Gal III and mock transfected cells occurred mainly at high molecular weight bands, which are likely to correspond to cell membrane glycoproteins, such as integrins or E-cadherin, among others.

### Expression of α2β1 integrin and E-cadherin in Capan-1 and MDAPanc-28 clones upon ST3Gal III transfection

Cell surface expression levels of α2β1 integrin and E-cadherin molecules were assessed in Capan-1 and MDAPanc-28 transfected clones by flow cytometry.

CP and C31 cells showed similar levels of α2 integrin subunit, as well as of β1 subunit (**Figure 2A**). We had previously described that the levels of α2 subunit found in the MDAPanc-28 model were extremely low compared to Capan-1 model [30], what precluded further analysis of the α2β1 integrin glycosylation pattern influence on collagen type 1 adhesion using the MDAPanc-28 cell model. The corresponding study was then conducted with CP and C31 cells.

**Figure 2:** Expression of α2 and β1 integrin subunits, and E-cadherin in Capan-1 and MDAPanc-28 clones. **A**. Representative flow cytometry histograms of β1 and α2 integrin subunits surface expression in CP and C31 cells. Secondary antibody controls, dotted. **B**. Representative flow cytometry histograms of E-cadherin surface expression in CP, C31, M34 and MP cells. **C**. E-cadherin content of total cell lysates (TCL) from CP, C31, MP and M34 was analyzed by Western blotting. Tubulin was used as loading control in each cell line.

Concerning cell surface E-cadherin expression, the results showed similar levels between CP and C31, as well as between M34 and MP cells, with mean fluorescence intensity (MFI) values of 65.5 and 61.9 for CP and C31 cells and of 107.7 and 109.5 for MP and M34 cells. MDAPanc-28 model exhibited higher E-cadherin levels than Capan-1 model with an average of 1.7-fold increase in the MFI values (**Figure 2B**). A further comparison of E-cadherin protein content was performed with TCL and Western blot, and no significant differences among the four cell lines were detected (**Figure 2C**).

ST3Gal III overexpression did not modify either α2β1integrin or E-cadherin protein expression in C31 and M34 cells; therefore these clones are good models to study the potential influence of the differential glycosylation in the function of these two membrane glycoproteins.

### CP and C31 cellular adhesion to type 1 collagen and migration through collagen coated transwells is dependent on α2β1 integrin expression

To evaluate whether α2β1integrin is the main contributor to type 1 collagen adhesion and migration in Capan-1 model, function-blocking monoclonal antibodies (mAb) against specific integrin subunits were used in adhesion and migration assays.

CP and C31cells previously incubated with mAbs against α2 or β1 subunits showed extremely significant reduced rates of adhesion to type 1 collagen in a 92% and 73% for CP; and in a 89% and 69% for C31, respectively (p<0.001); whereas mAbs against other important integrin subunits (α3, α5) did not change the adhesion rates significantly (**Figure 3A**).

**Figure 3:** Influence of α2β1 surface expression in the adhesion and migration of CP and C31 cells. Adhesion (**A**) and migration (**B**) of CP and C31 cells to type 1 collagen using mAbs against α2, α3, α5 or β1 integrin subunits or α2 or β1 integrin subunits, respectively. Bars represent mean ± SD. * Significantly different compared within the same cell line (p<0.05); ^#^ significantly different compared within CP and C31 cells (p<0.001).

Blocking of other receptors that could be involved in type 1 collagen recognition such as α1β1 integrin was not studied since Capan-1 has been reported to barely express this integrin [15], [16]. Likewise, neither α10β1 nor α11β1 integrins were studied due to their restricted expression in chondrocytes [37] and mesenchymal cells [38], respectively.

Migration assays through collagen coated transwells were performed with CP and C31 cells previously incubated with mAbs against α2 or β1 integrin subunits. Migration rates were significantly diminished, in a 66% and 46% for CP, and in an 81% and 68% for C31, respectively (p<0.001) (**Figure 3B**).

These results show the involvement of α2β1 integrin in the adhesion to collagen and migration in CP and C31. Since the same expression levels of α2 integrin subunit, as well as of β1, were found in C31 and CP cells (**Figure 2A**), next experiments were addressed to determine whether α2β1 integrin glycosylation was different between these clones and could thus explain the changes in adhesion and migration previously described [23], [30] and corroborated again in this study where C31 cells show lower adhesion to type 1 collagen and increased migration through collagen compared to CP cells.

### Differences in α2β1 integrin sialylation pattern between CP and C31 cells

Human α2 integrin subunit has 10 potential *N*-glycosylation sites, one of them (Asn-343) identified by mass spectrometry analysis [39], [40]; whereas β1integrin subunit has 14 potential sites, six of which (Asn-212, 403, 406, 411, 481 and 669) have also been identified [39], [40], [41]. To determine the SLe^x^ and α2,6-sialic acid content on α2β1 integrin molecules, biotinylated C31 and CP α2 integrin immunoprecipitate blots were analyzed with mAb against SLe^x^ and with SNA lectin.

Two typical bands for the α2 subunit at 170 kDa, and a band of approximately 120 kDa, which corresponds to the β1 subunit coprecipitated with α2, were detected. A slight increase of SLe^x^ staining on the α2 subunit of C31 cells, together with a major decrease of α2,6-sialic acid on both α2 and β1 subunits, compared to CP was found (**Figure 4A**; *upper panels*). Equivalent amounts of loaded protein were verified by reprobing the corresponding membranes with HRP-conjugated streptavidin, which in addition provided information of the α2 and β1 subunit levels (**Figure 4A**; *lower panels*). The blots also showed that α2,6-sialic acid is predominantly expressed on the coprecipitated β1 subunit, while SLe^x^ is basically found on the α2 subunit. The results lead us to conclude that the α2β1 integrin molecules of C31 cells show a much lower content of α2,6-sialic acid and slightly higher SLe^x^ levels than that of CP mock cells.

**Figure 4:** Sialylation of α2β1 integrin and FAK tyrosine 397 phosphorylation in CP and C31 cells. **A**. α2 integrin subunit immunoprecipitates from biotinylated cells were blotted and analyzed with mAb against SLe^x^ (*right upper panel*) or with *Sambucus nigra* agglutinin (SNA; *left upper panel*). Equivalent amounts of loaded protein were verified by reprobing the corresponding membranes with HRP-conjugated streptavidin. **B**. Lysates from cells plated onto type 1 collagen coated dishes or kept in suspension were blotted and incubated with mAb against phosphorylated tyrosine 397 FAK (pY397 FAK) and with mAb against total human FAK. Bands were quantified and the relative FAK Y397 phosphorylation per cell line was calculated as the quotient between pY397 FAK quantification and total FAK quantification (graph). Bars represent mean ± SD. * Significantly different (p<0.05).

### Overexpression of SLe^x^ induced alterations in intracellular signaling pathway derived from integrin-collagen binding

To address whether changes in α2β1 integrin glycosylation could affect the integrin-dependent signaling pathway, the autophosphorylation of focal adhesion kinase (FAK) at tyrosine 397 was analyzed. Both CP and C31 cells bound to collagen showed significant increased phosphorylation of FAK Y397 compared with CP and C31 kept in suspension, which showed lower levels of endogenous phosphorylation. Interestingly, relative Y397 phosphorylation levels in C31 cells bound to collagen raised 2.7-fold (p<0.001) compared with C31 cells in suspension, in a significantly higher degree (p<0.01) than the increase of Y397 phosphorylation in collagen bound CP cells compared with CP cells in suspension, which was of 1.7-fold (p<0.01) (**Figure 4B**). Since Y397 phosphorylation promotes cell motility through the formation of FAK/Src complex and the subsequent activation of different pathways related to cell migration [9], [42], the higher increase of FAK Y397 phosphorylation in C31 cells could, at least in part, contribute to explain the higher migration capacity of C31 compared to CP cells.

### ST3Gal III transfected cells showed decreased cell-cell aggregation and increased invasion capability

The role of the ST3Gal III sialylation on cell-cell aggregation and invasion capacity was assessed. A significant decrease in cell-cell aggregation of the ST3Gal III transfected cells compared to mock was shown after 24 h of cell seeding. MP cells formed 10-fold larger cellular aggregates than M34 (p<0.01), and CP cells formed about 3-fold larger aggregates than C31 (p<0.01). In general, Capan-1 model showed more disperse aggregates than MDAPanc-28 model (**Figure 5A**).

**Figure 5:** Aggregation on agar and Matrigel invasion assays. **A**. Representative microscopy images (40X) of cellular aggregates after 24 h of seeding the cells on soft agar coated wells. Mean particle size quantification in pixels (*right graph*). **B**. Invasion of CP, C31, MP and M34 cells through Matrigel coated inserts for 24 h. Bars represent mean ± SD. * Significantly different (p<0.01).

The invasive potential was assessed by *in vitro* invasion assay through Matrigel, which consists on a solubilized basement membrane-like preparation, mainly composed by laminin-111, collagen IV, heparan sulfate proteoglycan, various growth factors and additional components [43]. The results showed that Capan-1 model was around 6-times more invasive than MDAPanc-28 model (**Figure 5B**). Concerning ST3Gal III transfectants, there was a significant increase in the rate of cellular invasion when comparing to the corresponding controls cells. In particular, C31 cells exhibited 2.5-fold higher invasion rates than CP (p<0.001) and M34 cells were 3-fold more invasive with respect to MP (p<0.01). Interestingly, the described assay also measures the ability of the cells to attach to the ECM, invade into and through it, along with their migratory capacity toward a chemoattractant, crucial steps during the metastatic cascade [44], which were higher in the ST3Gal III transfectants.

### SLe^x^ and E-cadherin cellular expression in the ST3Gal III transfected pancreatic cancer cells

Immunofluorescence labeling of cell monolayers with mAbs against E-cadherin and/or SLe^x^ showed similar E-cadherin levels among ST3Gal III and mock transfected cells, as observed by western blot and flow cytometry analysis. However, a slight delocalization of this protein to the cytoplasm was observed mainly in the ST3GalIII transfected cells M34 and, to a lesser extent, in C31 cells (white triangles in **Figure 6**; *left column*) when compared to their corresponding mock cells.

**Figure 6:** E-cadherin and SLe^x^ immunolabeling in cell monolayers. Representative fluorescence microscopy images (400X) of E-cadherin (*left columnt*), SLe^x^ epitope (*mid column*) and merge (*right column*) in cell monolayers. Nuclei were stained with DAPI (blue). White triangles highlight areas of E-cadherin delocalization (left column) and areas of SLe^x^ and E-cadherin colocalization (right column). Close-up in inserts of E-cadherin localization are shown (630X).

As expected, a significant increase in SLe^x^ staining was detected in the ST3Gal III overexpressing clones of both cell models (**Figure 6**; *mid column*). Colocalization of E-cadherin and SLe^x^ at the cell membrane was shown in Capan-1 model (CP and C31) and also in M34 cells (white triangles in **Figure 6**; *right column*).

Morphological analysis revealed important differences in the cellular phenotype and in cell-cell contacts between both models and between the ST3 Gal III transfectants and their corresponding controls. MP cells grew in compact spherical aggregates with tight cell-cell adhesion and expression of E-cadherin at the cells membrane. Upon ST3Gal III transfection (M34), alteration of the cellular morphology was observed with cells showing a more disperse phenotype with loss of intercellular contacts concomitantly with delocalization of E-cadherin into the cytoplasm. CP and C31 cells, in their turn, showed stellate morphology with faint contacts among cells, and especially in C31 notable holes were present in the midst of the monolayer (**Figure 6**).

Although the protein levels of E-cadherin did not show significant differences among the four cell lines (**Figure 2B and 2C**), morphologic changes in cell-cell contacts with E-cadherin delocalization in the ST3Gal III transfected clones suggested a possible alteration of the adhesive function in these cells, which could contribute to explain their loss of cell-cell aggregation capacity and higher invasion.

To evaluate whether changes in SLe^x^ and/or α2,6-sialic acid determinants in the ST3Gal III transfected cells could occur on the E-cadherin molecule we analyzed the sialylation pattern of E-cadherin glycan chains.

### E-cadherin sialylation profile in the ST3Gal III transfected pancreatic cancer cells

*N-*glycosylation contributes up to 20% of E-cadherin total mass, and several reports support the involvement of *N-*glycans in the modulation of E-cadherin-mediated tumor cell-cell adhesion [25], [26], [27]. E-cadherin sialylation pattern was evaluated by immunoprecipitation followed by lectin blot analysis. E-cadherin from the four cell lines was detected at 120 kDa range, and its sialylation profile was analyzed using mAb against SLe^x^, and with SNA and MAL-II lectins, which detect α2,6-sialic acid and some α2,3- sialic acid determinants excluding SLe^x^ [45], respectively. SLe^x^ epitope could not be detected on E-cadherin (data not shown), whereas α2,3- and α2,6-sialic acid levels were faintly detected. To assess the changes in E-cadherin sialylation, the levels of sialic acid of each cell line were normalized with the corresponding E-cadherin levels. ST3Gal III transfected cells showed a slight decrease of α2,6-sialic acid levels compared to the corresponding controls, predominantly in the M34 clone (**Figure 7A**), together with an increase in α2,3-sialic acid determinants (**Figure 7B**).

**Figure 7:** E-cadherin sialylation status. Immunoprecipitation of E-cadherin followed by α2,6- or α2,3-sialylation recognition using *Sambucus nigra* agglutinin (**A**) or *Maackia amurensis* lectin II (MAL-II) (**B**) lectins, respectively.

Taken together, these differences in the overall sialylation, and in E-cadherin sialylation in particular, are in accordance with the observed changes on the cellular morphology and E-cadherin cellular distribution and function observed in the ST3Gal III transfected cells, and could account for the differences in *in vitro* cellular aggregation and invasion assays.

### E-cadherin, α2β1 integrin and SLe^x^ expression in human pancreatic ductal adenocarcinoma tissues

The expression of E-cadherin, α2β1 integrin and SLe^x^ molecules was evaluated in healthy pancreas and PDAC tissues from human patients (**Figures 8** and **9**). With regards to E-cadherin, healthy tissues displayed a strong and organized expression of E-cadherin at the cell contacts along the typical pancreatic acinus (**Figure 8**; *upper panel*), whereas PDAC samples showed clear disorganization of the tissue structure, along with the characteristic intense fibrotic response or desmoplasia. Moreover, in the tumor tissues a progressive delocalization of E-cadherin was observed, as well as loss of E-cadherin expression in a number of tumor cells in some of the samples (**Figure 8**; *lower panel*). Faint stain of α2 and β1 integrin subunits was found in the duct cells of healthy pancreas, and β1 integrin also stained the endothelial blood vessel cells (data not shown). In PDAC samples, higher expression of α2 and β1 subunits was found in the tumor cells and in the desmoplastic stroma (**Figure 9**). β1 subunit was also expressed by the endothelial cells (**Figure 9**; *lower panel*). *De novo* expression of SLe^x^ determinant was found in the tumor cells of PDAC tissues throughout the dense stroma (**Figure 8**; *lower panel* and **Figure 9**). Areas of SLe^x^ and E-cadherin colocalization were detected in the tumor areas (**Figure 8**; white arrows), and colocalization of α2 integrin subunit and SLe^x^ was found in a few tumor cells (**Figure 9**, white arrows). No colocalization of β1 subunit and **SLe^x^** could be detected.

**Figure 8:** Immunohistological study of SLe^x^ and E-cadherin expression in human PDAC tissues. Representative images (400X) of E-cadherin (green), SLe^x^ (red) and nucleus (blue) staining in human healthy and pancreatic ductal adenocarcinoma (PDAC) tissues from stages IIA and IIB. Whereas healthy tissues displayed a strong and organized expression of E-cadherin at the cell contacts, PDAC samples showed clear disorganization of the tissue structure and a progressive delocalization as well as loss of E-cadherin expression in a number of tumor cells. *De novo* expression of SLe^x^ is visible in every PDAC tissue. White triangles denote areas of SLe^x^ and E-cadherin colocalization.

**Figure 9:** SLe^x^ and α2 and β1 integrin subunits expression in human PDAC tissues. Representative images of merged immunofluorescence staining of α2 integrin (green, *upper panel*; 100X and 400X) or β1 integrin (green, *lower panel*; 200X and 400X) with SLe^x^ (red) and nucleus (blue) in pancreatic ductal adenocarcinoma (PDAC) tissues. α2 and β1 integrins are displayed in tumor cells. They also stain the stromal cells (indicated as D, for desmoplasia) and β1 integrin stains the endothelial cells of blood vessels (see arrow). SLe^x^ is found in the lumen of tumor cells and in some secretions. No colocalization of β1 integrin and SLe^x^ could be detected. White triangles indicate points of α2 subunit and SLe^x^ colocalization.

## Discussion

The local microenvironment provides tissues with extrinsic barriers to limit the outgrowth of tumors at the primary site. But as tumors evolve, these pressures drive the selection for traits that enable cancerous cells to by-pass them [46]. Dissemination of carcinomas from their original sites of development to distant organs in the body is the cause for the major part of cancer morbidity and mortality. Although the molecular mechanisms underlying the cellular changes that take place during the invasive process are still not fully understood, there is a general consensus that cell-cell and cell-matrix interactions have to be profoundly altered [2], [47]. In fact, homophilic cell adhesion and integrin signaling are among the core signaling pathways that are altered in most pancreatic cancers, including genetically altered genes such as E-cadherin and integrins [48].

In previous studies we have demonstrated the influence of sialic acid determinants in cell-ECM adhesion and in migratory processes of various human cancer models, including gastric cancer cells [49], [50], and in pancreatic Capan-1 and MDAPanc-28 cell lines and their stably ST3Gal III transfected clones, C31 and M34 [25], [31]. Specifically, cell surface α2,6-sialic acid levels correlated with higher cell adhesion to ECM components, such as collagen, fibronectin and laminin, which are important components of the tumor stroma, while higher α2,3-sialic acid levels favored migration and metastasis [23], [30].

In the present work we have evaluated whether ST3Gal III overexpression and the subsequent changes in the pattern of sialylation have a role in cell-cell adhesiveness and invasion in the MDAPanc-28 and Capan-1 pancreatic cancer cell lines. In addition, we have evaluated the impact of sialylation in the regulation of E-cadherin and α2β1 integrin functions.

The human pancreatic adenocarcinoma Capan-1 and MDAPanc-28 ST3Gal III transfected cells have been shown to exhibit a reduced cell-cell aggregation capacity and a high migration and invasion capability when compared with their respective mock cells, which is in agreement with our previous works reporting their increased migration through collagen and *in vivo* metastatic potential in mice [23], [30]. In addition, Capan-1 cells display higher expression of SLe^x^ levels than MDAPanc-28 cells, which consequently show a higher invasive potential and lower aggregation rates than MDAPanc-28. These results reinforce the importance of α2,3-sialic acid in potentiating cell invasion and metastasis. In accordance, major α2,3-sialic acid residue expression was associated with higher invasive and metastatic potential of gastric and breast cancer cells [50], [51], [52] and, conversely, decreased α2,3-sialic acid levels of a lung cancer cell model resulted in invasion and metastasis suppression [53]. Likewise, induction of a more invasive phenotype by the terminal glycan structures containing α2,3-sialic acid through the activation of invasion-related signaling pathways has been recently reported in gastric carcinoma cells [50].

Pancreatic adenocarcinoma is characterized by a particularly high desmoplasia [12], [54], and several studies have converged on the hypothesis that type 1 collagen plays an active role *in vitro* and *in vivo* in the pathophysiology of this neoplasia [15], [55]. Our results showed that adhesion to type 1 collagen and migration through this ECM protein is dependent on α2β1 integrin in CP and C31 cells, which is in agreement with other reports in pancreatic cancer cell lines [15]. Moreover, we have also shown that α2 and β1 integrins are expressed in the tumor cells and in the desmoplastic stroma of PDAC, in agreement with published studies that describe the expression of α2β1 integrin in pancreatic cancer cells and its interaction with type IV collagen in PDAC tissues [56].

Several studies have hypothesized that alteration on *N*-glycosylation may act as a regulatory mechanism for β1 integrins function [57], [58], [59]. The presence of *N*-glycans on the α5β1 heterodimer, which is the best-characterized integrin molecule, and on the β4 subunit has been reported to be crucial for proper integrin-ECM interactions [60], [61]. However, only the *N*-glycans localized in certain motifs are proposed to regulate the conformation and biological function of these glycoproteins, either facilitating the subunit association and/or regulating the integrin activation state [62]. In addition, the modification of integrin *N*-glycans by sialyltransferases enzymatic activity results in integrin subunits being capped with the negatively charged sugar sialic acid, which can modulate integrin function [63].

In our study we have shown that α2β1 integrin glycosylation was different between pancreatic cancer Capan-1 cells overexpressing ST3Gal III and mock cells. The results showed a slight increase in SLe^x^ glycans expression in the α2 subunit and a significant decrease in α2,6-sialic acid content in both α2 and β1 subunits of C31 cells. Since higher α2,6-sialic acid levels in pancreatic cancer cells correlated with increased ECM adhesion [30], we here suggest that the decrease in α2,6-sialic on the α2β1 integrin molecule appears to contribute for the reduced adhesion of C31 cells to type 1 collagen. This hypothesis is consistent with several reports stating that the downregulation of α2,6-sialyltransferase ST6Gal I inhibited cell adhesion to collagen and that, conversely, the hypersialylation of the β1 integrin subunit with α2,6-sialic acid promoted adhesion to collagen of several cancer cells [64], [65], [66]. C31 cells also showed a more migratory phenotype. Similarly, Guo et al. [34] described that human fibrosarcoma cells MGAT5 transfected, which showed reduced attachment to fibronectin due to glycosylation changes in their α5β1integrins, increased their migration.

Recent studies have demonstrated that SLe^x^ can be determinant for the behavior of cancer cells by modulating tyrosine kinase receptors [50]. In the present work we demonstrate for the first time the functional role of SLe^x^ in integrin mediated function. Here we show that the Capan-1 cells overexpressing ST3Gal III glycosyltransferase, C31 cells, display an enhanced SLe^x^ pattern of expression in general and particularly on the α2 integrin molecule compared with the CP control cells (**Figure 4A**), suggesting a regulatory effect of SLe^x^ on α2β1integrin-dependent migration. In PDAC tissues, α2 and β1integrin subunits were expressed in some of the tumor cells all over the cell surface. SLe^x^ antigen was also expressed in some tumor cells and was specially found at the ductal lumen and in foci of tumor cells, as largely described by other authors [21], [22], [67]. Although the pattern of staining of the integrin molecules and SLe^x^ antigen was different, some areas of α2 integrin and SLe^x^ colocalization were detected in a few tumor cells.

The importance of integrin glycosylation in the activation of FAK has been described by several authors. The level of FAK tyrosine phosphorylation was shown to be reduced in α1,6-fucosyltransferase (Fut8) deficient mouse embryonic fibroblasts [35], as well as in HeLa S3 cells transfected with β1,4-*N*-acetylglucosaminyltransferase (GnT-III) [68]. Likewise, a dependence on integrin sialylation has been reported for FAK/paxillin-mediated signaling, and for cancer angiogenesis and metastasis pathways [69]. In our Capan-1 clones, FAK Y397 was more highly phosphorylated in C31 than in CP upon binding to collagen, which contributes for a higher motility of C31, that is in agreement with previous reports describing that autophosphorylation of FAK Y397 is elevated in highly motile and invasive cancer cells [70]. Since the decrease of α 2,6-sialylation β1 integrin subunit has been reported to reduce tumor migration [71], we suggest that the increase of SLe^x^ in α2β1 integrin may favor the higher phosphorylation of FAKY397 upon collagen adhesion (**Figure 4B**), and therefore the more migratory and invasive phenotype of the human pancreatic adenocarcinoma cells C31 versus CP cells (**Figures 3B** and **5B**). In line with this, recent studies have described that changes in cell glycosylation may alter the cell phosphoproteome, and particularly the SLe^x^ overexpressing gastric cancer cells increase the phosphorylation of FAK Y397 and contributed to explain their higher invasive capacity [50].

Interestingly, we have further demonstrated that E-cadherin is a carrier of sialylation in the pancreatic cancer cell lines, being a target of modification by the ST3Gal III enzyme. In particular, an increase in α2,3-sialic acid and a decrease in α2,6-sialic acid was shown in the E-cadherin molecule of the ST3Gal III overexpressing cells. This specific modification of E-cadherin with terminal sialylated structures was concomitantly observed with alterations in cellular morphology together with alterations on E-cadherin cellular localization compared with control cells. In addition, these alterations could account for the observed decrease in cell-cell aggregation of the ST3Gal III transfectants together with their increased invasive potential. In PDAC clinical samples. E-cadherin expression was found in some tumor areas, with points of E-cadherin and SLe^x^ colocalization where a potential interface between both molecules could exist.

In conclusion, we have demonstrated that the alteration of the membrane sialylation pattern of PDAC cells has a modulatory effect in the proper function of important membrane adhesive molecules such as α2β1 integrin and E-cadherin, influencing cell adhesion and invasion processes. In particular, increase in SLe^x^ and decrease in α2,6-sialic acid as a consequence of ST3Gal III transfection led to reduced cell-cell adhesiveness, and endowed the cells with a more invasive phenotype. Glycosylation of E-cadherin and α2β1 integrin molecules was also modified as a result of the ST3Gal III transfection, with impact in the modulation of their functions and thus underlying the observed differences in the adhesive and motile phenotype. Specifically, glycan changes in α2β1 integrin of ST3Gal III transfected cells were further shown to activate integrin-mediated signaling pathways through FAK phosphorylation and therefore contributing to increase cell migration.
